This article has been retracted.

# An ECG Heartbeat Classification Method Based on Deep Convolutional Neural Network

**DOI:** 10.1155/2021/7167891

**Published:** 2021-09-27

**Authors:** Dengqing Zhang, Yuxuan Chen, Yunyi Chen, Shengyi Ye, Wenyu Cai, Ming Chen

**Affiliations:** ^1^Department of Cardiology, Jinjiang Municipal Hospital, Fujian, Jinjiang 362200, China; ^2^School of Informatics Xiamen University, Xiamen University, Fujian, Xiamen 361000, China; ^3^Department of Public Health, Jinjiang Municipal Hospital, Fujian, Jinjiang 362200, China

## Abstract

The electrocardiogram (ECG) is one of the most powerful tools used in hospitals to analyze the cardiovascular status and check health, a standard for detecting and diagnosing abnormal heart rhythms. In recent years, cardiovascular health has attracted much attention. However, traditional doctors' consultations have disadvantages such as delayed diagnosis and high misdiagnosis rate, while cardiovascular diseases have the characteristics of early diagnosis, early treatment, and early recovery. Therefore, it is essential to reduce the misdiagnosis rate of heart disease. Our work is based on five different types of ECG arrhythmia classified according to the AAMI EC57 standard, namely, nonectopic, supraventricular ectopic, ventricular ectopic, fusion, and unknown beat. This paper proposed a high-accuracy ECG arrhythmia classification method based on convolutional neural network (CNN), which could accurately classify ECG signals. We evaluated the classification effect of this classification method on the supraventricular ectopic beat (SVEB) and ventricular ectopic beat (VEB) based on the MIT-BIH arrhythmia database. According to the results, the proposed method achieved 99.8% accuracy, 98.4% sensitivity, 99.9% specificity, and 98.5% positive prediction rate for detecting VEB. Detection of SVEB achieved 99.7% accuracy, 92.1% sensitivity, 99.9% specificity, and 96.8% positive prediction rate.

## 1. Introduction

According to the latest World Health Statistics 2019 [1] report, heart disease, the top killer of humanity, was the primary cause of death worldwide in the past two decades, accounting for 16% of all causes of death. Since this kind of disease severely contributes to a lower life expectancy, the detection and diagnosis of cardiovascular diseases perform an inestimable value for all human beings. At present, some diagnostic methods, including ECG, ultrasonic cardiogram (UGC), chest X-ray, and cardiac Magnetic Resonance Imaging (MRI), are extensively used to detect cardiovascular diseases. Specifically, the ECG plays a significant part among these measures due to its affordable and convenient superiority. ECG signals are the most popular way to monitor the health status of the cardiovascular system and identify diseases related to the cardiovascular system. The morphological changes of the electrocardiogram and the depolarization of the myocardium can be profitable to assist in the diagnosis of heart disease. However, the complex ECG data makes manual identification a challenge, which demands the rich experience of doctors. Considering this, many scholars have applied various algorithms to help detect these diseases, improving the classification model in accuracy, speed, and robustness. Many popular methods, such as decision trees, random forest, and SVM, are proposed in ECG data classification. Many scientists have researched popular machine learning algorithms and neural network algorithms, proving that the latter is effective for heart disease classification, with higher credibility and slighter error. These neural networks can learn relationships and information that are difficult for people to discover from a large amount of complex data.

As manual analysis is time-consuming, laborious, and easy to misjudge, this paper refers to VGGNet [2], designing an ECG arrhythmia classification model based on CNN. We classify and learn ECG data thoroughly and aim to improve accuracy by building and optimizing neural networks. In our paper, the ECG dataset is divided into five categories to realize a rough assessment of the heart state, providing an essential and reliable reference for the doctor's further diagnosis. The proposed method is used to classify based on all datasets. The results show that our classifier achieved an average accuracy of 99.76%, an average sensitivity of 94.45%, an average specificity of 99.54%, and an average positive prediction rate of 97.40%. Moreover, to evaluate the proposed model, we compared the results of other deep learning algorithms to detect VEB and SVEB, and the proposed method obtained better results.

## 2. Literature Review

Many scientists have conducted related researches on the classification of ECG data. Houssein et al. [3] presented a new morphological features descriptor and proposed a method based on a metaheuristic algorithm termed Manta ray foraging optimization (MRFO) and SVM, obtaining 98.26% accuracy and 97.43% sensitivity. Mathunjwa et al. [4] converted 1D ECG signals into 2D segments, combined recurrence plot (RP) and CNN to make arrhythmia classification, and achieved the accuracy of 95.3% on ventricular fibrillation (VF) categories and 98.41% on the atrial fibrillation (AF), normal, premature AF, and premature VF categories. Pirova et al. [5] compared random forest, decision tree, and convolutional neural network algorithms, showing that the neural network is superior to other algorithms in ECG data classification, with an accuracy rate of 93.47%. Baloglu et al. [6] proposed an end-to-end deep learning model based on standard 12-lead ECG signals to diagnose myocardial infarction. They used a deep CNN model, which completed the ECG signal learning process at the end of a short period (10 epochs). Furthermore, manually extracting features from the original ECG data or using the features learned by other machine learning models is unnecessary with this method. Jun et al. [7] put forward a deep two-dimensional convolution method to classify ECG data and converted every ECG beat into a two-dimensional grey-scale image as the input data of the classifier. Their CNN-based ECG arrhythmia classification consists of two steps: ECG and data preprocessing. At the same time, they applied methods such as batch normalization, data enhancement, and Xavier initialization to optimize the CNN classifier, and the average accuracy rate was up to 97.85%. This result convinced that the use of ECG images and the CNN model to detect arrhythmia is effective.

Furthermore, various machine learning algorithms are widely used. Methods such as support vector machines (SVM) have been tested to classify ECG arrhythmia detection. Kohli et al. [8] compared three popular SVM algorithms, one-against-one, one-against-all, and fuzzy decision function, and finally concluded that the one-against-one method performs better results when distinguishing the cardiac arrhythmia and grouping them into the correct class. Considering that the artificial neural network (ANN) has the flaw of converging to a local minimum and is prone to overfitting, Walsh [9] used the support vector machine algorithm to classify the ECG data as it tends towards an optimal margin separation, as the search space constraints define a convex set. However, due to the imbalance of the data, the support vector machine macroaverage F1 score only reached 0.87.

In addition, as a commonly used classification algorithm, KNN is also applied to classify ECG data. Saini et al. [10] used it as a classifier to detect QRS waves of ECG signals. The detection rate of the CSE DS-3 MIT-BIH arrhythmia database is 99.89% and 99.81%, proving the effectiveness and reliability of KNN. The ECG signal was decomposed by wavelet transform to improve efficiency, and thirteen (including energy feature) statistical features were evaluated from these decomposed signals by Saini et al. [11]. The classification efficiency of the decomposed ECG signals was increased by 31.25% to 87.5%.

Besides, Kanani et al. [12] were concerned about the importance of data preprocessing, introducing a preprocessing technique used for ECG classification that significantly improves the accuracy and stability of the training models. Through data preprocessing, the system's accuracy can reach more than 99% without overfitting. Huang et al. [13] apply the cardiovascular disease electronic health framework based on IoT devices with wearable sensors, which can effectively and timely treat patients with cardiovascular disease.

## 3. Materials

### 3.1. ECG Database

In this paper, we apply the MIT-BIH arrhythmia dataset [14, 15], which is famous for assessing arrhythmias and applied for the fundamental analysis of cardiac dynamics. With the annotation of at least two cardiologists, this database contains excerpts from 48 and a half hour double-channel recordings. Gained by the BIH Arrhythmia Laboratory, these recordings were obtained from 47 testers from 1975 to 1979. Each contains two 11-bit resolution ECG lead signals in the 10 mv range, digitized at 360 samples per second. In compliance with the Association for the Advancement of Medical Instrumentation (AAMI) EC57 standard [16], these annotations were grouped into five different categories. To understand the mapping between different categories and descriptions and AAMI EC57 categories, refer to Table 1.

### 3.2. Convolutional Neural Network

The convolutional neural network is a feedforward neural network with a deep structure, and it is the most widely used algorithm for deep learning [17, 18]. It has the characteristics of multilevel network structure, no complicated preprocessing, partial connection, and shared weights. The three main convolutional neural network architecture layers are the convolutional, pooling, and fully connected layers.

The convolutional layer is the core layer of the neural network, composed by sliding the incompatible convolution kernel on the input matrix and running certain operations. A neuron in the convolutional layer is connected to only one neuron in the local window of the previous layer to form a local connection network. The convolution kernel only captures specific local features in the input data. Therefore, to extract multiple features, we need to use multiple different convolution kernels.

Pooling is a significant step in CNN, which is also called the subsampling layer. Max pooling divides the input data into several rectangular areas and outputs the maximum value for each subarea, reducing the number of neurons.

The fully connected layer plays a vital role in classifying the network, and each neuron is fully connected to all neurons in the upper layer. As shown in Figure 1, due to the effect of full connection, the parameters of the weight matrix will significantly increase. On the contrary, the convolution layer adopts a local connection. With the same color connection, the weight is the same, and the number of parameters of the final weight matrix will be significantly reduced.

## 4. Methodology

In this paper, we designed a CNN-based ECG arrhythmia classification method. The method has the following steps: ECG data preprocessing, model training, and model evaluation. We preprocessed the MIT-BIH arrhythmia database and divided the preprocessed five types of ECG data into mutually exclusive training sets and test sets for training and testing the CNN classifier. We used the training set to train the CNN classifier, and after getting the relevant training model, it is used to predict the classification of the 5 ECG types in the test set. The overall process of the method in this paper is shown in Figure 2.

### 4.1. Data Preprocessing

The dataset was preprocessed with a method proposed by Kachuee et al. [19], and we achieve good results by inputting the processed ECG data directly into the neural network we built. The process of data preprocessing proposed is as follows:

1. *Normalization.* Select a specific 10 s window of ECG signal and normalize the amplitude to be in the range of 0 to 1.
2. *Find the R-Peak Candidates of ECG Data.* Applying a threshold of 0 : 9, the R-peak candidate set is selected from the local maximum of normalized data.
3. *Select the Signal.* For each r-peak, a signal with a length of 1.2 times the median of R-R time intervals is selected and paddled with zeros to satisfy a predefined fixed length.

After the original signal is processed, it is classified into five different ECG signals. After processing, we divide the data into the training and test sets, including the 87554 and 21892 test sets. Each data is part of the electrocardiogram, expressed as a vector of 187 values.  Table 2 shows the distribution of datasets in different categories after preprocessing.

### 4.2. Apply Flattening to the Network

Because the output of the convolutional and pooling layers is two-dimensional, the data needs to be flattened. Then the result obtained by the convolutional layer is input to the fully connected layer. It follows that we use the fallen layer for transition between the convolutional layer and the fully connected layer, which converts the multidimensional results obtained by the convolutional layer to one dimension and inputs them into the fully connected layer. To summarize, the output of the convolutional layer is flattened to create a single long feature vector, as shown in Figure 3, and connected to the final classification model in the fully connected layer.

### 4.3. Apply the ELU Activation Function

The function of the activation function is to introduce nonlinear characteristics into the neural network model. In this paper, we mainly compare two nonlinear activation functions that are widely used in modern CNN models, including rectified linear unit (ReLU) and exponential linear unit (ELU) [20]. ReLU is one of the most commonly used activation functions in CNN. When the input is positive, there will be no gradient saturation problem. Moreover, there is only a linear relationship, so the calculation speed is faster than sigmoid and tanh. However, it will convert the negative input to zero, which will cause some neurons to stop participating in changes in the neural network. ELU solves this dying ReLU problem and retains the advantages of ReLU. ELU is an exponential function when the input is negative, and its overall output value is around zero, which is more robust.

The functions of ReLU and ELU are as follows:

(1) $$\begin{array}{c} \text{ReLU}\left(x\right)=\left\{\begin{array}{cc} 0, & \text{if }\left(x\leq 0\right),\\ x, & \text{if }\left(x>0\right), \end{array}\right)\\ \text{ELU}\left(x\right)=\left\{\begin{array}{cc} \alpha \left(e^{x}-1\right), & \text{if }\left(x<0\right),\\ x, & \text{if }\left(x\geq 0\right), \end{array}\right) \end{array}$$

where the value of the hyperparameter (*α*) is 1.0.

### 4.4. Optimized Classifier Architecture Similar to VGGNet

Given the above, we designed a CNN-based ECG arrhythmia classifier whose main structure is similar to VGGNet.  Figure 4 shows a schematic of the proposed network.  Table 3 describes the detailed architecture table of the proposed network. The proposed network contains 11 hidden layers, including nine one-dimensional convolutional layers and two fully connected layers. In this paper, kernel sizes of 3 and stride 2 are used in all convolutional layers, and all pooling layers use max pooling of size 2 and stride 2.

The mapping relationship between the heartbeat category and the heartbeat waveform is complicated [21], and we believe that single-layer convolution cannot complete the classification task well. Therefore, we use a coupled-convolution structure, two convolution layers, to get a better fitting effect. Furthermore, the use of deep convolution similar to the VGGNet framework can effectively improve the classification effect.

Most importantly, we used ELU as the activation function. We applied the TensorFlow open-source software library [22] to train and verify the model in the experiment. For network training, we used Adam optimizer [23] to optimize the parameters, where the learning rate is 0.001, beta-1 is 0.9, and beta-2 is 0.999, and used sparse categorical cross-entropy as the loss function.

In addition, to prevent overfitting of the model, we added Dropouts [24, 25] after the convolutional layers C2, C4, C6, and C9. Dropout randomly resets the weights of some neurons to 0 during each training process, reducing the number of parameters and avoiding overfitting.

### 4.5. Assessment Indicators

To evaluate the performance of the model, quantitative evaluation indicators are necessary. To this end, we applied four criteria to evaluate the classification effect of the CNN classifier proposed in this study, including accuracy (Acc), sensitivity (Sen), specificity (Spe), and positive prediction rate (Ppr).

The calculation formulas of the four indicators are as follows:

(2) $$\begin{array}{c} \text{Acc}=\frac{\text{TP}+\text{TN}}{\text{TP}+\text{TN}+\text{FP}+\text{FN}}\times 100,\\ \text{Sen}=\frac{\text{TP}}{\text{TP}+\text{FN}}\times 100,\\ \text{Spe}=\frac{\text{TP}}{\text{TP}+\text{FP}}\times 100,\\ \text{Ppr}=\frac{\text{TP}}{\text{TP}+\text{FN}}\times 100, \end{array}$$

where TP denotes true positive, FP denotes false positive, TN denotes true negative, and FN denotes false negative.

## 5. Results and Discussion

Based on all samples, we used the proposed method to classify and evaluate the ECG arrhythmia classifier.  Table 4 shows the confusion matrix of the classifier on all samples, and Table 5 shows the coefficients of the CNN method on all samples. Summarizing these data, we have less than 1% of ECG heartbeats misclassified in the experiment. Moreover, our proposed method achieved 99.76% average accuracy, 94.45% average sensitivity, 99.54% average specificity, and 97.40% average positive prediction rate based on all samples. Therefore, it is reasonable to believe that our proposed classifier can accurately predict and classify ECG arrhythmia signals.

Furthermore, we compare the proposed classifiers' performance with some other published methods based on evaluation indicators. Some studies only used part of the data from the MIT-BIH database, so it cannot be directly compared with the proposed method. For example, Jun et al. [7] excluded seven types of ECG arrhythmia from the MIY-BIH database, and only eight were classified.

Table 6 compares the VEB and SVEB classification performance of the proposed method with the other methods. The comparison experiments are based on the same dataset, which is intended to compare the classification performance of different classification methods. As it can be seen from this table, the proposed CNN classifier has excellent performance. The main reason behind this might be the fact that a network architecture similar to VGGNet is used. Research shows that network depth has an essential role in the classification effect [2]. All convolutional layers use smaller convolution kerVGGnels, which reduce the parameters and reduce the amount of calculation. It is worth mentioning that Shaker et al. [30] used Generative Adversarial Networks (GANs) equalization to process the dataset, making the model positive prediction rate slightly higher than the proposed model.

Additionally, by using a smaller convolution kernel to deepen the depth of the network and an activation function that accompanies each convolution layer, more activation functions can be added to have richer features and stronger dialectics. The classification accuracy of multiple small convolutions stacked is better than a single large convolution. In addition, we also selected ELU as the activation function, used the flattening layer to connect the convolutional layer and the fully connected layer, and used dropout to prevent overfitting. These works are also important reasons for obtaining good results.

During the experiment, we use dropout to prevent overfitting. Dropout is divided into a learning phase and a testing phase. In the learning phase, some hidden nodes will be temporarily ignored with a certain probability *p*, and the neural network will learn the local features in the data. In this way, feature learning in multiple simple networks can improve the generalization ability of the network. In the testing phase, the phases involved in learning and the hidden phase are summed with a certain probability p-weighted, and the network output is obtained by comprehensive calculation. Dropout can also be regarded as a kind of ensemble learning [31].  Figure 5 shows the loss and accuracy changes of training and verification steps when the epoch is 50. It can be seen from Figure 5 that the loss and accuracy curves of the verification step show a trend close to the training curve, and there is no gradual upward trend. Therefore, it is reasonable to conclude that the proposed model is not overfitting.

## 6. Conclusion

In this paper, we proposed a CNN-based ECG arrhythmia classification method. The ECG records of the MIT-BIH arrhythmia database are preprocessed and used as model input data. Finally, the trained model classified the ECG signal into five beats: normal beat, supraventricular ectopic beat, ventricular ectopic beats, fusion beat, and unknown beat. The optimized CNN model is designed with a network architecture similar to VGGNet using ELU activation function, dropout, and other technologies. According to the results, our proposed method performs well in the four-finger VEB and SVEB classification, with an overall average accuracy rate of 99.76%, which could accurately classify ECG signals. In recent years, data enhancement has attracted attention in ECG arrhythmia classification. Our future work aims to use data enhancement technology and various deep learning optimization techniques to classify arrhythmia better.

## Figures and Tables

**Figure 1:** Schematic diagram of convolutional neural network: (a) convolutional layer and (b) fully connected layer.

**Figure 2:** The proposed overall process of arrhythmia classification.

**Figure 3:** Schematic diagram of flattening layer.

**Figure 4:** Architecture of the proposed CNN classifier.

**Figure 5:** The (a) loss and (b) accuracy changes in training and verification steps.

**Table 1:** Mapping between different categories and descriptions and AAMI EC57 categories.

Category	Descriptions	Annotations
*N*	Nonectopic beat	Normal (NOR)
		Left bundle branch block (LBBB)
		Right bundle branch block beat (RBBB)
		Atrial escape (AE)
		Nodal (junctional) escape (NE)
*S*	Supraventricular ectopic beat	Atrial premature (AP)
		Aberrated atrial premature (aAP)
		Nodal premature (NP)
		Supraventricular premature (SP)
*V*	Ventricular ectopic beat	Premature ventricular contraction (PVC)
		Ventricular escape (VE)
*F*	Fusion beat	Fusion of ventricular and normal (fVN)
*Q*	Unknown beat	Paced (P)
		Fusion of paced and normal (fPN)
		Unclassifiable (U)

**Table 2:** Distribution of datasets in different categories after preprocessing.

Category	*N*	*S*	*V*	*F*	*Q*	Total
Train data	72471	2223	5788	641	6431	87554
Test data	18118	556	1448	162	1608	21892
Total	90589	2779	7236	803	8039	109446

**Table 3:** The structure of the proposed CNN classifier.

	Type	Biases	Kernel size	Stride	Output size
Layer 1	Convolution	16	3	1	(185, 16)
Layer 2	Convolution	16	3	1	(183, 16)
Layer 3	Max pooling	—	2	2	(91, 16)
Layer 4	Convolution	32	3	1	(89, 32)
Layer 5	Convolution	32	3	1	(87, 32)
Layer 6	Max pooling	—	2	2	(43, 32)
Layer 7	Convolution	64	3	1	(41, 64)
Layer 8	Convolution	64	3	1	(39, 64)
Layer 9	Max pooling	—	2	2	(19, 64)
Layer 10	Convolution	128	3	1	(17, 128)
Layer 11	Convolution	128	3	1	(15, 128)
Layer 12	Convolution	128	3	1	(13, 128)
Layer 13	Max pooling	—	2	2	(6, 128)
Layer 14	Flatten	—	—	—	(768)
Layer 15	Fully connected	30	—	—	(30)
Layer 16	Fully connected	5	—	—	(5)

**Table 4:** Confusion matrix of CNN method on all samples.

	Predicted					
Ground truth		*N*	*S*	*V*	*F*	*Q*
	*N*	90447	80	30	24	8
	*S*	199	2559	19	0	2
	*V*	74	3	7123	31	5
	*F*	83	1	58	661	0
	*Q*	33	0	3	0	8003

**Table 5:** Coefficients of the CNN classifier for classification of all samples.

Category	Acc (%)	Sen (%)	Spe (%)	Ppr (%)
*N*	99.51	99.84	97.94	99.57
*S*	99.72	92.08	99.92	96.82
*V*	99.80	98.44	99.89	98.48
*F*	99.82	82.32	99.95	92.32
*Q*	99.95	99.55	99.99	99.81
Average	99.76	94.45	99.54	97.40

**Table 6:** Comparison of VEB and SVEB classification performance of the proposed method with other methods.

Methods	Classifier	VEB				SVEB			
		Acc	Sen	Spe	Ppr	Acc	Sen	Spe	Ppr
Jiang et al. [26]	BBNN	98.8	94.3	99.4	95.8	97.5	74.9	98.8	78.8
Kiranyaz et al. [27]	1D-CNN	99.0	93.9	98.9	90.6	97.6	60.3	99.2	63.5
Acharya et al. [28]	DA + CNN	97.9	94.2	98.8	95.3	97.0	90.6	98.6	94.3
Zhai et al. [29]	2D-CNN	99.1	96.4	99.5	96.4	97.3	85.3	98.0	71.8
Shaker et al. [30]	GAN + CNN	99.5	94.5	99.7	98.6	99.1	91.2	99.3	97.7
**Proposed**	**1D-CNN**	**99.8**	**98.4**	**99.9**	**98.5**	**99.7**	**92.1**	**99.9**	**96.8**

BBNN: block-based neural networks, 1D: one-dimensional, 2D: two-dimensional, CNN: convolutional neural networks, DA: data augmentation, and GAN: generative adversarial networks.

## Data Availability

The website for obtaining the MIT-BIH arrhythmia database is https://www.physionet.org/content/mitdb/1.0.0/, and the preprocessed ECG database is obtained from the website: https://www.kaggle.com/shayanfazeli/heartbeat.
